# Bone Mineral Density Prediction from CT Image: A Novel Approach using ANN

**DOI:** 10.1155/2023/1123953

**Published:** 2023-04-28

**Authors:** S. L. Resmi, V. Hashim, Jesna Mohammed, P. N. Dileep

**Affiliations:** Department of Mechanical Engineering, TKM College of Engineering, Kollam, Kerala, India

## Abstract

**Background:**

Though treatable, osteoporosis continues as a substantially underdiagnosed and undertreated condition. Bone mineral density (BMD) monitoring will definitely aid in the prediction and prevention of medical emergencies arising from osteoporosis. Although quantitative computed tomography (QCT) is one of the most widely accepted tools for measuring BMD, it lacks the contribution of bone architecture in predicting BMD, which is significant as aging progresses. This paper presents an innovative approach for the prediction of BMD incorporating bone architecture that involves no extra cost, time, and exposure to severe radiation.

**Methods:**

In this approach, the BMD is predicted using clinical CT scan images taken for other indications based on image processing and artificial neural network (ANN). The network used in this study is a standard backpropagation neural network having five input neurons with one hidden layer having 40 neurons with a tan-sigmoidal activation function. The Digital Imaging and Communications in Medicine (DICOM) image properties extracted from QCT of human skull and femur bone of rabbit that are closely associated with the BMD are used as input parameters of the ANN. The density value of the bone which is computed from the Hounsfield units of QCT scan image through phantom calibration is used as the target value for training the network.

**Results:**

The ANN model predicts the density values using the image properties from the clinical CT of the same rabbit femur bone and is compared with the density value computed from QCT scan. The correlation coefficient between predicted BMD and QCT density valued to 0.883. The proposed network can assist clinicians in identifying early stage of osteoporosis and devise suitable strategies to improve BMD with no additional cost.

## 1. Introduction

Osteoporosis is a progressive, systemic, and skeletal disease which is characterized by low bone mass and microarchitectural deterioration of bone tissue, leading to increased bone fragility and consequent increase in fracture risk [1]. The peak bone mass at young adulthood depends largely on genetic, biological, and lifestyle factors, since low bone strength during the growing years is evidently associated with increased fragility fracture risk during old age [2]. It is reported that bone loss starts from the age of 30–40 years in both men and women [3]. In women, marked increase in bone loss during premenopause and postmenopause is observed, while in men a small longitudinal bone loss is seen throughout life [4, 5]. A worldwide estimate shows that one in three women as well as one in five men, above the age of 50 years, will experience osteoporotic fractures and may lead to decreased quality of life and increased medical costs [6]. Moreover, it is testified that 50 million people in India are either osteoporotic or have low bone mass conditions, making the disease a major health concern in the region [7]. With the progression of osteoporosis, the stress induced on the vertebrae as well as deformation on intervertebral disk increases under various body postures [8]. Studies evaluated that the osteoporotic bone might have been adapted to lower load level than high or sudden loads [9]. Also, it is reported that when nonhabitual error loads were applied, stress and strain in the osteoporotic vertebrae were much higher than those in healthy ones [10]. Eighty-four percent of osteoporotic fracture cases are due to ignorance of worsening of bone mass [11].

Though osteoporosis is incurable, it remains markedly underdiagnosed and inadequately treated. Hence, early detection of impaired quality of bone is crucial in the prevention of osteoporotic fracture and helps in starting timely bone modulating therapies. Bone mineral density (BMD) plays a major role in evaluating the osteoporotic condition of a patient. The measurement of BMD is significant in diagnosing and therapy monitoring of osteoporosis as well as to predict fracture risk.

Dual-energy X-ray absorptiometry (DEXA) of total hip, femoral neck, and lumbar spine is the most widely used tool for diagnosing osteoporosis. It is reported that DEXA scan provides defective diagnosis due to the involvement of cortical bone which can be a source in overestimation of BMD [12]. Additionally, DEXA scan includes posterior element of the spine leading to inaccurate prediction in case of severe spinal degeneration and in scoliosis patients. Many researchers have used quantitative computed tomography (QCT) as a tool for measuring BMD [13]. The BMD value can be measured with minimum error using QCT due to the fact that superposition of cortical bone and other tissues seldom occurs and the results are expressed in milligrams per cubic centimeter of calcium hydroxyapatite. This is unique among various clinical methods for assessing bone density because it can be used to quantify the spatial distribution of density in three dimensions [14]. Possible exposure of the patient to radiation and associated high cost are considered as its drawback. Moreover, greater amount of time and technical expertise are required to deduce BMD values using QCT.

Recently, osteoporosis is being predicted from *T*-score derived through CT attenuation number (Hounsfield units (HU)) from clinical CT images [12]. Even though routine clinical CT is less expensive and is widely used for diagnostic purposes in various medical disciplines, this method of osteoporosis prediction using CT attenuation number lacks clinical support as compared to DEXA [15]. But, *T*-score based on DEXA score is not accurate in majority of patients who sustain fragility [12]. From the above discussions, it can be envisaged that osteoporotic diagnosis using the predicted BMD from patient-specific CT images can replace the prediction method like DEXA which is expensive with high radiation exposure. Many researchers have demonstrated that microstructure and mechanical properties of bone can be derived from texture analysis of CT images [16]. Furthermore, research has shown that calculating three-dimensional (3D) Haralick texture measures from low-resolution CT scans can help predict bone microarchitecture [17]. It is reported that incorporating bone architecture can improve the bone density predictability to 90% [18]. Two-dimensional (2D) projection of the bone images can be utilized to measure texture features. Texture information related to trabecular structure is conserved during the transformation from 3D to 2D images using software analysis [19]. Studies establish that texture features like energy, entropy, correlation, contrast, and homogeneity show good correlation to bone mechanical properties [20]. The routine clinical CT examination images that are taken for other indications can be used for a one-step prediction of BMD values, and then the osteoporotic diagnosis can be achieved with no additional cost, patient time, equipment, and software or radiation exposure. Differential measurements of local variations, such as co-occurrence matrices or gray-level run length approach, are two statistical texture analysis methods that can be utilized for bone texture analysis. Haralick demonstrated that the gray level co-occurrence matrix (GLCM), which is a matrix with a number of rows and columns equal to the number of gray levels, G, in the image, is a popular method of extracting second-order texture information [21].

The GLCM quantitatively measures the frequency of different combinations of pixel brightness values occurring in an image. Each element in the matrix represents the position of pixels in the image having similar gray level values. The matrix element *P*(*i*, *j*|*d*, *θ*) is the relative frequency with which two pixels, one with intensity *i* and the other with intensity *j*, separated by a pixel distance (*d*) and at a particular angle (*θ*), occur within a given neighborhood. It is reported that 14 textural features can be measured from the probability matrix to extract the characteristics of texture statistics of images and out of which the texture features such as angular second moment (energy), contrast, correlation, entropy, and the inverse difference moment (homogeneity) have good correlation with mechanical properties of bone [17, 20–22]. Hence, in this study, these five texture features are selected as the input parameters of artificial neural network (ANN) for predicting the BMD.

ANN is a system that simulates the human brain which is suited for solving nonlinear problems [8, 23]. ANN is an effective data information system with the ability to identify relationships from complex datasets and predict outcomes. It consists of an input layer, an output layer, and one or more hidden layer with processing units termed as neurons which mimic the biological neurons. Among the various training algorithms, backpropagation learning algorithm minimizes the error function significantly in weight space using the method of gradient descent [24, 25]. The adaptive learning capability makes ANN model a powerful tool for data analysis and predictions [26, 27]. The application of ANN in the prediction of BMD and morphometric vertebral fractures in postmenopausal cases have been reported by many researchers [25–29]. In another study, ANN was used to predict future BMD and bone loss rate based on statistical data like age, weight, height, age at menopause, age at menarche, duration after menopause, body mass index (BMI), and so on [30]. It is also reported that ANN was used to diagnose osteoporosis more effectively and accurately, using micro-CT images by building a classifier for distinguishing osteoporosis and normal groups [31]. Though ANN was effectively used by these researchers for the diagnosis of osteoporosis, they have depended on statistical data from a wide range of topological features of the patients as the database for training the ANN and prediction of osteoporosis condition.

According to the authors' knowledge, no study has been published that employs image properties generated from the GLCM of a routine clinical CT scan taken for other purposes to predict osteoporosis using ANN. Through this paper, the authors intent to propose an ANN model developed for direct prediction of BMD from the second-order texture properties of a Digital Imaging and Communications in Medicine (DICOM) image of a routine clinical CT scan of an individual patient. In comparison to current methods that use topological properties of a patient, the proposed approach, if implemented, can be used to assess osteoporosis with high accuracy and at no additional expense.

## 2. Materials and Methods

Figure 1 shows the algorithm used in the present work for the prediction of BMD from routine clinical CT images. The BMD prediction algorithm consists of four major stages. In the first stage, QCT and clinical CT images of rabbit femur bone were acquired from GE Optima QCT Scanner having a phantom calibration—Catphan and Siemens CT scanner, respectively.

In the second stage, the GLCM matrix is formulated from DICOM images and five second-order texture properties such as energy, contrast, correlation, entropy, and homogeneity are estimated. The BMD values are extracted from the QCT images which are computed from the HU of the scan image through phantom calibration. The third stage trains the ANN model using the dataset which consists of five texture properties and the HU values extracted from the QCT. The QCT images of human skull supplied by Amrita Hospital, Ernakulam, were also used for training the network. In the final stage, the trained ANN is used to predict the BMD values using the texture properties extracted from clinical CT images.

The stepwise procedure of sample preparation and data acquisition for training and testing the network are discussed in the following sections.

### 2.1. Specimen Preparation

Femur bone specimens of adult rabbit weighing ∼1.75–2.5 kg are used for this study. Published methods for storage and handling of bone specimens were strictly followed during this investigation [32]. The specimens were kept at −20°C in saline solution until tested, thawed at room temperature, and kept moist with saline soaked sponge when prepared for QCT and clinical CT scans. Ethical approval was obtained from the University Ethics Committee (IAEC 1-KU-14/2019-20-TKM-PND (1)).

### 2.2. CT Images of Specimen

The dataset used for training the neural network is gathered from the QCT scanning (120 kV, 347 mA, 0.625 mm slice thickness) conducted on 15 rabbit femur bone specimens prepared as per the procedure reported by Ahmed and Voort [33]. The training data matrix is further populated with QCT image property data of human skulls which is supplied by Amirta Hospital, Ernakulam, India. The dataset used for testing the neural network is extracted from the QCT and clinical CT (120 kV, 347 mA, 1 mm slice thickness) images of nine rabbit femur bone specimens.  Figure 2 shows the sample DICOM image of rabbit bone. The target value for the neural network is the BMD value of each specimen which is extracted from the QCT image of the specimen using a tissue characterization phantom as a base reference to relate the BMD with the HU.

### 2.3. Define Region of Interest

The QCT and clinical CT images obtained are analyzed for identifying bone tissues or region of interest (ROI) by calculating tissue distribution from the mean gray value or HU value. This is done by using a ROI tool in the software Sante-DICOM Viewer. The selected ROI of an image is saved as jpeg image.  Figure 3 shows the selected ROI from the sample DICOM image with mean/standard deviation (SD) of gray value.

### 2.4. Feature Extraction from Selected Region of Interest

Energy, entropy, contrast, homogeneity, and correlation, which quantify the spatial relationship between pixels in the area under investigation (ROI), had the best correlate with BMD [17]. The GLCM values with orientations 0°, 45°, and 90° for a displacement of one unit for the selected ROI unit were extracted from the QCT images of rabbit bone and human specimens. The texture parameters are computed from average GLCM values using MATLAB code. Using MATLAB code, second-order texture metrics extracted from GLCM, such as energy, entropy, contrast, homogeneity, and correlation, are used as ANN inputs.

The parameter energy (*E*_*n*_) measures the number of repeated pairs in the image. It is computed as the sum of squares of entries in the GLCM and is given by:

(1) $$\begin{array}{c} E_{n}=\sum_{i=0}^{Ng-1}\sum_{j=0}^{Ng-1}P_{ij}^{2}, \end{array}$$

where *i*, *j* are the spatial coordinates of the function *P*(*i*, *j*) and Ng is the gray tone of the image.

The parameter entropy (*E*_t_) measures the randomness of gray level distribution within the image and is given by:

(2) $$\begin{array}{c} E_{t}=\sum_{i=0}^{\mathrm{Ng}-1}\sum_{j=0}^{\mathrm{Ng}-1}-P_{ij}\times \log\;P_{ij}. \end{array}$$

The parameter contrast (Co) measures the local variations present in an image and is defined as:

(3) $$\begin{array}{c} Co=\sum_{i=0}^{N-1}\sum_{j=0}^{N-1}{\left(i-j\right)}^{2}P\left(i,j\right). \end{array}$$

The parameter homogeneity (Ho) measures the uniformity of image and is defined as:

(4) $$\begin{array}{c} \mathrm{Ho}=\frac{\sum_{i=0}^{Ng-1}\sum_{j=0}^{Ng-1}P_{ij}}{1+{\left(i-j\right)}^{2}}. \end{array}$$

The parameter correlation (*C*) property measures the linear dependency of gray levels of neighboring pixels and is given as:

(5) $$\begin{array}{c} C=\frac{\sum_{i=0}^{Ng-1}\sum_{j=0}^{Ng-1}\left(i,j\right)p\left(i,j\right)-\mu_{x}\mu_{y}}{\sigma_{x}\sigma_{y}}, \end{array}$$

where, *μ*_*x*_*μ*_*y*_ and *σ*_*x*_*σ*_*y*_ are the mean gray tone values and standard deviation of gray tone values, respectively.

The formulation of GLCM and computation of the five second-order texture properties from the saved ROI of QCT and clinical CT image was computed using MATLAB code. These textures properties constitute the training set of the ANN and a sample dataset for training the network is shown in Table 1.

### 2.5. Artificial Neural Network (ANN) Analysis

The network used in this study is a standard backpropagation neural network, which consists of an input layer, an output layer, and a hidden layer. The input layer of the network contains five neurons that receives texture features, such as energy, contrast, correlation, entropy, and homogeneity, which are extracted from the DICOM image. The output layer contains only one neuron which gives the predicted BMD value. A layer with 40 neutrons as a hidden layer and the tan-sigmoidal function as the activation function are used in this work.

The activation function decides whether a neuron will activated or not. The value of neuron in a feedforward neural network is calculated as:

(6) $$\begin{array}{c} Y=\sum_{i=1}^{m}\left(x_{i}\times w_{i}\right)+b, \end{array}$$

(7) $$\begin{array}{c} \text{tan}h\left(x\right)=\frac{2}{1+e^{-2x}}. \end{array}$$

The tan-sigmoid (tan*h*) activation function has strong gradient and big learning steps. The output of tan*h* is symmetric around zero leading to faster convergence.

The network architecture used in this study is given in Figure 4 and is implemented using MATLAB code.

The dataset used for training the neural network includes 300 sets of five texture features as the input data and the corresponding BMD values extracted from QCT images as the target data. The training dataset is extracted from QCT images of 15 rabbit femur bone and human skull specimens supplied by Amrita Hospital, Ernakulam. The five texture features extracted from these scanned images are used as input data and the corresponding density value of the bone which is computed from the HU of the QCT scan image through phantom calibration is used as the target data for training the network.

During the training phase, the network uses 70% of dataset for training, 15% of dataset for validation, and the remaining for testing the network. Upon converging, the accuracy of the trained network is further established using the texture properties extracted following routine clinical CT images captured from the nine rabbit femur bone samples.

## 3. Result and Discussion

This work mainly focused on the prediction of BMD values from clinical CT images taken for other indications using neural network.

There are works reported on deriving BMD from microstructural analysis of bone [16]. Moreover, early works established that clinical CT image quality is sufficient to analyze second-order image properties [17]. Also, studies correlated bone microstructure, bone volume/total volume (BV/TV), trabecular spacing, trabecular thickness, and trabecular number strongly with second-order texture properties [34]. In a feedforward network, each layer's neurons are only connected to the neurons in the following layer. The backpropagation (BP) supervised learning technique is used in current feedforward network to dynamically change the weight and bias values for each neuron in the network. The network is trained using the dataset extracted from the QCT images of 15 rabbit bone samples and human skull supplied by the Amrita Hospital, Ernakulam. The texture properties are extracted from a specific region, namely, the ROI of bone. In this work, 300 ROIs are used for extracting the image properties.

The training dataset contains the BMDs extracted from the QCT images of rabbit specimens and human skull. The density values extracted from the image vary from 0.9 to 1.87 g/cm^2^. Sample dataset is shown in Table 1. The scatter plot of training dataset is shown in Figure 5(a)–5(e). The proposed ANN is subjected to training using the training dataset and the network is converged with a learning rate of 0.19 after four epochs. The strength of linear relationship between predicted output and the target output is computed using the correlation coefficient (*R*) and is plotted against the predicted and target BMD values (Figure 6).

It may be noted from Figure 6(a)–6(c) that the correlation coefficient between the target BMD and the neural network predicted BMD values for training, validating, and testing datasets are 0.9878, 0.9245, and 0.9501, respectively. An overall correlation coefficient of 0.9715 has been obtained, as shown in Figure 6(d), indicating a very good agreement with predicted BMD and those values obtained from QCT during training phase which indicates convergence during ANN training.

The above results reveal that the proposed ANN, after training, shows excellent capability to predict BMD as compared to the density extracted from QCT images. The mean squared error (MSE) of 0.19043, from the validation performance graph, also indicates a very good agreement in the predicted values of density. All curves, as shown in Figure 7, converges to a single point showing that the network performed equally well in training, validation, and testing phases.

The accuracy of the trained network is further established using the matrix of texture properties extracted from the clinical CT images of nine rabbit femur bone specimens. The BMD values extracted from the QCT images of the same samples were depended for comparison. It is noted that the predicted BMD values of the rabbit femur bone specimens from the routine clinical CT image properties using the trained neural network are well within 90% as against the BMD values computed from QCT images.  Figure 8 shows that the correlation coefficient between QCT computed BMD and predicted BMD from clinical CT is 0.9027. Hence, the proposed approach can be used as a simple method for the determination of BMD using routine clinical CT scan images taken for other indications. This novel approach will open a safe and cost-effective way for prediction of osteoporotic conditions.

## 4. Conclusion

In this study, an approach based on image processing and ANN for predicting BMD from clinical CT image is presented. The network used in this study is a standard backpropagation neural network, which consists of an input layer with five neurons, an output layer with one neuron, and a hidden layer with 40 neurons. The five inputs are the texture properties such as energy, entropy, correlation, homogeneity, and contrast extracted from CT images and the output is BMD. The dataset used for training the neural network includes 300 sets of five texture features as the input data and the corresponding BMD values as the target data, extracted from QCT images of rabbit femur bone specimens and human skull supplied by Amrita Hospital, Ernakulam, India. The overall correlation coefficient for the training phase valued to 0.9715 indicates that the trained ANN model is converged and can predict BMD values.

To the best of knowledge, no studies in predicting BMD from clinical CT image have been reported; however, the BMD computed from QCT has been compared with predicted values of the current network, as shown in Figure 8. The accuracy of the proposed network is established using the dataset from clinical CT images of rabbit femur bone specimens and noted that the predicted BMD values of the rabbit femur bone specimens from the routine clinical CT image properties using the trained neural network are well within 90% as against the BMD values computed from QCT image. The ANN proposed in this paper demonstrated that BMD values can be predicted using the texture features extracted from clinical CT image taken for any diagnostic purposes. The proposed methodology will assist clinicians in identifying early stages of osteoporosis and devise suitable strategies to improve BMD without additional radiation exposure and cost incurred during specific diagnosis of osteoporosis.

### 4.1. Limitation and Future Scope of the Work

The methodology limits the training dataset to human skull bone and rabbit femur. This work can be extended and generalized by considering bone image data (training data) in a wider age group, incorporating gender, bone images from varying human habitat.

## Figures and Tables

**Figure 1:** Overview of the four-stage bone mineral density prediction from clinical CT images.

**Figure 2:** Sample DICOM image of rabbit bone.

**Figure 3:** 2D image with mean/SD of gray value.

**Figure 4:** Schematic view of the neural network architecture developed.

**Figure 5:** Scatter plot of training dataset: (a) entropy, (b) contrast, (c) energy, (d) homogenity, and (e) correlation.

**Figure 6:** Comparison between bone mineral density from QCT and ANN predicted values for the (a) training dataset, (b) validation dataset, (c) test dataset, and (d) overall performance.

**Figure 7:** Validation performance graph between number of epochs and mean squared error.

**Figure 8:** Scatter plot shows the correlation between predicted BMD from clinical CT and BMD computed from QCT.

**Table 1:** Sample dataset for training the network.

Input dataset					Output dataset
Contrast	Correlation	Energy	Homogeneity	Entropy	Bone mineral density
3	0.6936	0.5454	0.8889	2.7036	1.89847
3.3667	0.6639	0.3489	0.8722	3.9166	1.909341
5	0.6124	0.44	0.8333	3.5435	1.785716
5.05	0.5284	0.425	0.8083	3.2676	1.681617
5.25	0.5493	0.4514	0.8056	3.0029	1.686442
3.5	0.6576	0.5216	0.8704	2.7869	1.844213
5.5	0.4952	0.4883	0.8021	3.3537	1.897391
0.6	0.8589	0.4816	0.8817	2.7931	1.726328
6.6875	0.3527	0.2344	0.6302	3.3842	1.70792

## Data Availability

No data were used to support this study.
